RETRACTED

# miR-551b regulates epithelial-mesenchymal transition and metastasis of gastric cancer by inhibiting ERBB4 expression

**DOI:** 10.18632/oncotarget.17392

**Published:** 2017-04-24

**Authors:** Guangyuan Song, Hongcheng Zhang, Chenlin Chen, Lijie Gong, Biao Chen, Shaoyun Zhao, Ji Shi, Ji Xu, Zaiyuan Ye

**Affiliations:** ^1^ The Second Clinical Medical College, Zhejiang Chinese Medical University, Hangzhou, Zhejiang, China; ^2^ The First Clinical Medical College, Zhejiang Chinese Medical University, Hangzhou, Zhejiang, China; ^3^ Department of Gastrointestinal and Pancreatic Surgery, Zhejiang Provincial People's Hospital, Hangzhou, Zhejiang, China; ^4^ Key Laboratory of Gastroenterology of Zhejiang Province, Hangzhou, Zhejiang, China

**Keywords:** miR-551b, epithelial-mesenchymal transition (EMT), metastasis, gastric cancer, ERBB4

## Abstract

Epithelial-mesenchymal transition (EMT) is an important biological process that is characteristic of malignant tumor cells with metastatic potential. We investigated the role of miR-551b in EMT and metastasis in gastric cancer (GC). We found that low miR-551b levels were associated with EMT, metastasis and a poor prognosis in GC patients. Further, two GC cell lines, MNK45 and SGC7901, exhibited lower miR-551b levels than the GES normal stomach cell line. Exposing MNK45 and SGC7901 cells to TGF-β1 resulted in cell morphology changes characteristic of EMT, which was confirmed by Western blot analysis demonstrating low E-Cadherin and high N-Cadherin and Vimentin levels. Treatment with miR-551b mimics inhibited these EMT changes as well as Transwell migration and invasiveness. We identified ERBB4 as a potential target of miR-551b based on patient data from the TCGA. ERBB4 was upregulated in GC specimens, and its high expression correlated with a poor prognosis of GC patients. Dual luciferase assays revealed that miR-551b directly inhibited ERBB4 by binding to its 3′UTR. Moreover, treatment with miR-551b mimics or the ERBB4 inhibitor AST-1306 inhibited EMT in the GC cell lines. Finally, nude mice xenografted with GC cancer cell lines expressing miR-551b mimics exhibited smaller tumors and longer survival than mice engrafted with control GC cancer cells. These data indicate that miR-551b inhibits EMT and metastasis in GC by inhibiting ERBB4. miR-551b and ERBB4 are thus potential therapeutic targets for the treatment of GC.

## INTRODUCTION

Gastric cancer (GC) has the highest morbidity and mortality rates in the world, especially in China [1]. The most common method of GC treatment is surgery, which has a high success rate when diagnosed early [2]. However, most patients are diagnosed when the cancer has already metastasized. The high metastasis rate and low chemotherapy sensitivity result in poor survival rates among GC patients [3, 4]. Therefore, suppression of metastasis is the key to improve the survival rate of GC [5].

RETRACTED

MicroRNAs (miRNAs) are a class of endogenous non coding small RNAs that play an important role in many physiological processes [6–8]. miRNAs are generally 22-24 nucleotides long and complementary to mRNA 3′ non-coding region, thereby inhibiting the translation or negatively regulating transcription of target genes [9–11]. Most importantly, microRNAs regulate various stages of tumor development and progression including proliferation, apoptosis and multi-drug resis-tance [9, 12–16]. miR-551b is known to regulate the malignant behavior of GC [17]. Due to the low expression of miR-551b in GC tissue, it is postulated to function as a tumor suppressor [18]. However, the specific role and mechanism of miR-551b in the metastasis of GC is unclear. Therefore, we conducted both *in vitro* and *in vivo* experiments to investigate the molecular mechanism of miR-551b in inhibiting metastasis and EMT of GC.

## RESULTS

### miR-551b is down-regulated in gastric cancer

We analyzed the miRNA-seq data from 21 gastric cancer samples obtained from The Cancer Genome Atlas (TCGA) datasets to identify critical miRNAs involved in gastric cancer. The heat map analysis showed that miR-551b was significantly downregulated in the tumor tissues compared to the normal stomach tissues (Figure 1A and 1B). Further, qRT-PCR analysis showed that miR-551b was significantly decreased in MNK45 and SGC7901 gastric cancer cell lines compared to immortalized stomach GES cells (Figure 1D). For further confirmation, miR-551b levels were quantified in 27 frozen gastric cancer specimens paired with adjacent normal tissues. Again, the expression of miR-551b was significantly lower in tumor tissues than the matched adjacent normal tissues (Figure 1C). Further analysis demonstrated that low miR-551b levels in TCGA gastric cancer data was closely related to the poor survival rate of GC patients suggesting that miR-551b was a prognostic indicator of GC (Figure 1E).

**Figure 1:** miR-551b is down-regulated in gastric cancer **(A)** Heat map analysis of the miRNA profiles for the 21 gastric cancer cases from the TCGA database using R software (P_adj_ <0.05 and log_2_ fold change >3) is shown. **(B)** miR-551b expression between normal and tumor samples is plotted from the heat map. **(C)** Fold expression of miR-551b in normal and tumor tissues are shown. **(D)** RT-PCR analysis of miR-551b expression (fold) in GES, MNK45 and SGC7901cells is shown as mean ± SD. Note: ** is *P* < 0.01. **(E)** Plot shows the percent survival rate of GC patients with high (red) and low (blue) expression of miR-551b. High expression of miR-551b is associated with long term survival.

RETRACTED

### miR-551b inhibits invasion and migration of GC cell lines *in vitro*

Since miR-551b levels were low in the MNK45 and SGC7901 gastric cancer cells, we treated the cells with miR-551b mimic to generate cells with significantly enhanced miR-551b levels (Figure 2) and compared the consequences using *in vitro* invasion and migration assays. Towards this, we compared control and miR-551b-mimic transfected MNK45 and SGC7901 cells in invasion and Transwell migration assays 24h after treatments. We observed that cells transfected with the miR-551b mimic showed significant reduction in migration and invasion (Figure 3A-3D). This suggested that miR-551b inhibited GC metastasis.

**Figure 2:** Fold expression of miR-551b in control or miR-551b mimic treated SGC7901 (left) and MNK45 (right) cells is shown ** *P* < 0.01.

**Figure 3:** miR-551b significantly inhibits invasion and migration of **(A)** MNK45 and **(B)** SGC7901 cells treated miR-551b mimics compared to the control. **, p < 0.01. DAPI stained images (100x) of miR-551b mimic transfected **(C)** MNK45 and **(D)** SGC7901 cells (right) compared to control group (left) demonstrating inhibited invasion (top) and migration (bottom) are shown.

### miR-551b inhibits the EMT induced by TGF-β1

Since miR-551b mimics inhibited invasiveness and metastasis of GC cell lines *in vitro*, we wanted to study the effects of miR-551b on the epithelial to mesenchymal transition (EMT) that confers metastatic ability to tumor cells. Towards this, we treated the MNK45 and SGC7901 cells with 10ng/ml TGF-β1 (TGF-β1 is a classical inducer of cell EMT) for 24h and observed the changes in cell morphology under a microscope (Figure 4E). We observed that the cells changed from quadrilateral to spindle shape with rich and long microfilament tentacles that demonstrated the ability to migrate and invade (Figure 4A-4C). Further, Western blotting data showed that E-Cadherin was reduced and N-Cadherin and Vimentin increased in cells treated with TGF-β1 that was characteristic of EMT. In contrast, cells treated with miR-551b mimic demonstrated quadrilateral shape and no characteristic microfilament organization along with enhanced E-Cadherin and reduced N-Cadherin and Vimentin levels that suggested inhibition of EMT (Figure 4D and 4F). These results suggested that TGF-β1 induce EMT in gastric cancer cells and miR-551b inhibited EMT.

**Figure 4:** miR-551b mimics inhibit EMT induction by TGF-β1 in gastric cancer cell lines Images (200x) showing morphological changes in MNK45 and SGC7901 cells show extensive filipodia and lamellipodia in untreated cells **(A, B, C** and **E)** compared to TGF-β1 treated cells. **(D** and **F)** Western blot analysis showing changes in E-Cadherin, N-Cadherin and Vimentin levels in control, control treated with TGF-β1 and miR-551b mimic plus TGF-β1 treated MNK45 and SGC7901 cells. β-actin was used as internal control.

RETRACTED

### ERBB4 is the target of miR-551b

To identify the putative targets of miR-551b, the TargetScan was performed and 3′-UTR of ERBB4 mRNA was recognized as the potential target of miR-551b (Figure 5A). The dual-luciferase reporter assay was used to validate if ERBB4 was a direct target of miR-551b. We observed that co-transfection of miR-551b mimics significantly enhanced the luciferase activity of the ERBB4 3′-UTR reporter, but, the luciferase activity of ERBB4 reporter with mutated miR-551b binding sites remained basal (Figure 5D-5G). This suggested that miR-551b specifically targeted ERBB4. Further, we quantified the expression of ERBB4 in 27 pairs of frozen GC tissue specimens with their adjacent normal tissues and again observed that the expression of ERBB4 was significantly higher in tumor tissues than in normal tissues (Figure 5B). Moreover, ERBB4 was associated with the survival rate of GC patients based on the analysis TCGA data (Figure 5C). Together, these results strongly suggest that ERBB4 promotes EMT and metastasis in GC based on its regulation by miR-551b.

**Figure 5:** ERBB4 is a direct target of miR-551b **(A)** Sequence alignment of miR-551b with the 3′ UTR of ERBB4 and the mutated miR-551b binding site are shown. **(B)** The mRNA expression of ERBB4 in normal and tumor tissues is shown. **(C)** Survival curve of GC patients from the TCGA database showing the relationship between expression of ERBB4 and patient survival time. **(D-G)** Dual luciferase reporter assay comparing control amd miR-551b mimic treated MNK45 and SGC7901 cells in presence of wild type or mutated ERBB4 UTR is shown. **, p < 0.01.

### Correlation between ERBB4 and EMT

Further, to study the correlation between ERBB4 and EMT, we stained MNK45 and SGC7901cells with anti-ERBB4 antibody and TRICTC conjugated Phalloidin for actin cytoskeleton (Figure 6A-6D). We observed that the GC cells that showed high expression of ERBB4 demonstrated stretched lamellipodia and filopodia characteristic of EMT cells. Compared to the control cells (Figure 6D, red box), the expression of ERBB4 in the EMT cells was higher (Figure 6D, arrows). Western blot analysis demonstrated that treatment with ERBB4 inhibitor AST-1306 resulted in increased E-Cadherin and reduced N-Cadherin and Vimentin in both MNK45 and SGC7901 cells, similar to miR-551b mimic transfected cells (Figure 6E and 6F). This suggested that ERBB4 was critical for EMT in GC.

RETRACTED

**Figure 6:** ERBB4 expression regulates EMT in MNK45 cells induced by TGF-β1 **(A)** Immunoflorescence staining with anti-ERBB4 antibody. **(B)** Cytoskeleton staining: of MNK45 cells induced by TGF-β1 were stained by TRITC conjugated Phalloidin. **(C)** Nuclear DAPI staining of GC cells induced by TGF-β1. **(D)** Merge of A-C Red arrows point to EMT cells showing stretched out lamellipodia and filopodia and enhanced cytoplasmic expression of ERBB4. The red box shows cells with low ERBB4 expression with non-EMT characteristics. The images shown are under 200x magnification. **(E** and **F)** Inhibition of EMT due to ERBB4 inhibition by AST-1306 in MNK45 and SGC7901 cells by Western blot analysis of E-Cadherin, N-Cadherin and Vimentin are shown. β-actin was used as internal control.

### miR-551b regulates ERBB4 translation

We further explored the mode of miR-551b regulation of ERBB4 by analyzing the effect of miR-551b mimics on mRNA and protein expression levels of ERBB4. We observed by RT-PCR that ERBB4 mRNA levels in both the MNK45 and SGC7901 cells that were transfected with miR-551b mimics were comparable to the negative controls (Figure 7A and 7B). However, Western blot analysis showed that treatment with miR-551b mimics downregulated ERBB4 protein levels (Figure 7C and 7D). This suggested that miR-551b regulated ERBB4 translation and not at the transcriptional level.

**Figure 7:** miR-551b regulates ERBB4 translationally **(A and B)** Relative levels of ERBB4 mRNA in untreated and miR-551b mimic treated MNK45 and SGC7901 cells based on RT-PCR is shown. **(C and D)** Western blot analysis of ERBB4 protein in untreated and miR-551b mimic treated MNK45 and SGC7901 cells is shown.

### miR-551b supresses tumor growth *in vivo* and prolonged the survival time

Finally, to confirm the anti-tumor effects of miR-551b *in vivo*, we used a xenograft mouse model. First, MNK45 and SGC7901 cells were transfected with either miR-551b-mimics or control and then injected into the subcutaneous or peritoneum of nude mice. The tumor sizes were measured every 7 days for 5 weeks and the tumor growth was visualized by the animal living imaging system (PerkinElmer, USA). Our analysis demonstrated that control cells formed significantly larger tumors than the miR55b mimic transfected cells in the nude mice, both in case of subcutaneous and peritoneal injections (Figure 8A and 8B). Further, the tumor volume was significantly diminished in case of miR-551b mimic treated cells compared to the control cells (Figure 8C). Most importantly, miR-551b mimic treated cells resulted in significantly enhanced survival time of tumor bearing nude mice (Figure 8D).

RETRACTED

**Figure 8:** Xenograft mouse model shows that miR-551b mimics significantly inhibit tumor growth and extend life span **(A and B)** Live imaging of subcutaneous and peritoneal tumor growth at 14 days in untreated (left) and miR-551b mimic treated GC cells (right) demonstrating that miR-551b diminishes tumor growth in nude mice. **(C)** Tumor volume curve showing growth of untreated and miR-551b mimic transfected GC cell tumors over a period of time (5 weeks). **(D)** Comparison of survival curves of nude mice injected with GC cells that are either untreated (blue) or transfected miR-551b mimic (red) are shown.

## DISCUSSION

GC is among the most common malignant cancers and currently ranks second for most morbidity and mortality cases worldwide [1]. Most patients are diagnosed when the tumor has already metastasized and therefore the benefits of surgery are restricted for many patients [19, 20]. Also, the invasion and metastasis of GC is critical to determining the survival time of patients after operation [21] with EMT preceding metastasis [22–24]. In this study, we demonstrated that miR-551b significant inhibited EMT, invasion and metastasis of GC cells. Further, miR-551b was significantly downregulated in GC tissues. Therefore, we postulated that miR-551b had tumor suppressor function based on our comparative analysis of GC cell lines MNK45 and SGC7901 with normal stomach cell line GES. Our data was corroborated by the analysis in GC patient samples demonstrating miR-551b was downregulated in advanced tumor samples and its expression correlated with GC patient survival time. Based on *in vitro* transwell migration and invasion assays, we demonstrated that miR-551b mimic treated MNK45 and SGC7901 cells were inhibited significantly in migrating through the matrigel, further suggesting that miR-551b inhibited tumor invasion and metastasis.

EMT is an important biological process that tumor cells undergo to become more invasive and metastatic [25–27]. We demonstrated that miR-551b inhibited EMT transition when the miR-551b mimic treated MNK45 and SGC7901 cells compared to control cells, based on cellular morphology as well as E-Cadherin versus N-Cadherin and Vimentin protein levels. By analyzing the TCGA data and clinical samples, we demonstrated that ERBB4 was a target of miR-551b; ERBB4 was overexpressed in GC tissues and significantly associated with the survival of GC patients. Further, immunofluorescence staining of ERBB4 combined with cytoskeletal staining suggested that high expression of ERBB4 correlated positively with EMT. Therefore, higher ERBB4 expression resulted in malignant GC (including EMT process, invasion and metastasis) and miR-551b negatively regulated ERBB4 expresssion.

RETRACTED

In summary, miR-551b regulates EMT and GC metastasis by inhibiting the expression of ERBB4 that significantly correlates with poor survival time. Thus, our data points that miR-551b is a potential prognostic factor and a therapeutic target for gastric cancer.

## MATERIALS AND METHODS

### Patients and tissue specimens

GC tumor tissues with matched adjacent non-tumor tissues were obtained from 21 patients that underwent surgical treatment at Zhejiang Provincial People's Hospital, (Hangzhou, Zhejiang, China). None of the patients had a history of chemotherapy or radiotherapy before sampling, and the diagnosis of GC was pathologically confirmed. This study was approved by the institutional ethic committee of Zhejiang Provincial People's Hospital, (Hangzhou, Zhejiang, China). All patients provided informed consent for this study.

### Cell culture

MNK45 and SGC7901 cells that were obtained from Shanghai cell bank (Chinese Academy of Sciences, Shanghai, China) were cultured in RPMI-1640 (Hyclone, Los Angeles, USA) containing 10% FBS (Gibco, MD, USA) at 37°C and 5% CO2.

### miR-551b mimic transfection

SGC7901 or MNK45 cells (1×10^5^ per well) were grown in a 6-well plate overnight followed by transfection with miR-551b mimics with Lipofectamine 2000 (Beyotime Biotechnology, Hangzhou, China), according to manufacturer's instructions. The miR-551b mimics were synthesized by GenePharma (Shanghai, China) and the negative control was purchased from RiboBio Co. Ltd (Guangzhou, China) for all experiments.

### Quantitative real-time PCR

To assess the transfection efficiency of the miR-551b mimics, qRT-PCR was performed using primers that were designed and synthesized by Sangon Biotech Ltd (Shanghai, China). The forward and reverse primers for miR-551b were 5′-ACACTCCAGCTGGGCTGAAACCAAGTATGGGTCG-3′ and 5′-TGGTGTCGTCGAGTCG-3′, respectively. The forward and reverse primers for U6 (control) were 5′-CTCGCTTCGGCAGCACA-3′ and 5′-AACGCTTCACGAATTTGCGT-3′, respectively. The total RNA of cells was extracted for reverse transcription. Then, cDNA was fully mixed with the designed primers and mixed enzymes. The PCR conditions were as follows: 95°C for 6 min, followed by 45 cycles of 95°C for 10 sec, 60°C for 60 sec and 72°C for 10 sec. Relative expression of miR-551b was calculated by the ΔΔCq method.

### Western blot analysis

Cells or tissues were lysed with cold lysis buffer (150mM NaCl, 1%NP-40, 1% Sodium deoxycholate, 0.1%SDS, 25mM Tris-HCl pH7.6) supplemented with protease inhibitor mixture (Beyotime Biotechnology, Hangzhou, China). The total protein concentration was measured using the BCA assay. Proteins were separated after constant voltage 110V electrophoresis for 90 minutes in SDS-PAGE gel, transferred electrophoretically onto nitrocellulose membranes at 300 mA current transfer for 90 minutes, and the protein bands were quantified using the gel imaging analysis system. Antibodies against β-actin, Vimentin, E- and N-Cadherin, were purchased from CST (MA, USA).

RETRACTED

### *In vitro* tumor cell migration and invasion assays

The Transwell assays (Corning, Cambridge, MA, USA) were performed to assay the migration of the GC cell lines. Briefly, cells were seeded into upper chamber and RPMI-1640 with 10% FBS was added in the lower chamber for 24h. Then, the cells on the upper surface of the membrane were removed by cotton swabs and the cells that migrated across the matrigel membrane were fixed with 10% methanol and stained with (2-(4-Amidinophenyl)-6-indolecarbamidine dihydro chloride, DAPI). Images were obtained with a fluorescence microscope (Nikon, Tokyo, Japan). For tumor cell invasion assays, the polycarbonate membrane was coated with matrigel and assays similar to Transwell migration assays described above were performed. All experiments were repeated thrice.

### *In vitro* EMT assays

MNK45 and SGC7901 cells were seeded in a 6-wells plate for 12h, followed by incubation with 10ng/ml recombinant human TGF-β1 (R&;D, Minneapolis, MN, USA) in RPMI-1640 for 24-48h. Proteins were then extracted from each group of cells and the EMT biomarkers, E-Cadherin, N-Cadherin, and Vimentin were detected by Western blot.

### Immunofluorescence assay

MNK45 and SGC7901 cells were seeded in a 6-wells plate with glass slides at the bottom. The cells were fixed with 4% paraformaldehyde for 15 minutes followed by permeabilization with 0.1% TritonX-100 for 1-5 minutes. Then, the cells were incubated with 1%BSA for 1h followed by overnight incubation with the anti-ERBB4 antibody (Cell Signaling Technology, Boston, USA) followed by the secondary antibody (Cell Signaling Technology, Boston, USA) and TRITC conjugated phalloidin (Sigma, MO, USA) for 30-60 minutes at room temperature. After staining with DAPI for 1-5 minutes at room temperature, fluorescence images were visualized with a laser scanning confocal microscope. Western blot analysis was also used to confirm the correlation between ERBB4 and EMT

### Dual luciferase reporter assay

Transcription factor-binding sites in the promoter region of human miR-551b were predicted by TargetScan and PicTar4 biological analysis website: http://www.targetscan.org and http://www.pictar.org. The putative ERBB4-binding site was 5′-AUGGGUCGA-3′, and the mutant ERBB4-binding site was 5′-UGUUUGAU-3′. The ERBB4 luciferase reporter constructs were made by amplifying the human ERBB4 mRNA 3′-UTR sequence by PCR and then cloning it into the XbaI site of the pGL3-promoter construct. The sequences of the human miR-551b promoter region were inserted into pGL3-basic vector (Sangon Biotech, Shanghai, China). The plasmids were then co-transfected with Renilla luciferase expression vector (pRL-TK) into MNK45 cells by Lipofectamine 2000 (Beyotime, Hangzhou, China) according to the manufacturer's instructions. After transfection for 24h, the luciferase activity was measured in samples by Dual-Luciferase Assay Kit (Beyotime, Hangzhou, China).

RETRACTED

### Xenograft mouse model

To examine the effect of miR-551b on the growth and metastasis of tumor cells *in vivo*, GC cell lines, SGC-7901 and MNK45 were transfected with luciferase vector (Sangon Biotech, Shanghai, China) with or without miR-551b mimic. Then, control and miR-551b mimic transfected MNK45 or SGC7901 cells (2×10^7^/ml) were injected with 100μl peritoneally or subcutaneously into nude mice and the tumor growth/volume was followed every 7 days for 5 weeks. To determine the tumor growth *in vivo*, the mice were injected with the NIRF dye (IR-783) into the vein after 7 days and the fluorescent signal was analyzed using the animal living imaging system (PerkinElmer, USA). The rate of tumor growth in the two groups of mice was plotted and analyzed. Also, Kaplan-Meier survival curves were used to analyze the effects of miR-551b mimics on the mice survival.

### Statistical analysis

The statistical analysis of data was performed with the SPSS 19.0 statistical software. The data were expressed as mean ±standard deviation; P<0.05 and P<0.01 were considered statistically significant
